# Oral Hygiene Habits and Use of Fluoride in Developmental Age: Role of Parents and Impact on their Children

**DOI:** 10.1155/2022/6779165

**Published:** 2022-07-11

**Authors:** Nicola Pranno, Giulia Zumbo, Martina Tranquilli, Luigi Stamegna, Francesca Zara, Iole Vozza

**Affiliations:** Department of Oral and Maxillo-Facial Sciences, Sapienza University of Rome, Rome, Italy

## Abstract

**Introduction:**

In healthcare, the need to pay more attention to the achievement of two objectives within the society arises: health promotion and prevention in terms of nutrition, good education, sport, and health education. Scientific evidence shows that adequate health standards must be learned since childhood through the help of parents and appropriate school projects. Parental intervention must be appropriate to support the responsibility of their children's health. In oral health, it has been established for many years that there is a correlation between parental behaviors and lifestyles and children's attitude. The aim of this study is to verify the close relation between behaviors, habits, lifestyles, and the knowledge of parents about their oral health and, consequently, their focus and care for their own children's oral health. Furthermore, the awareness of parents about the importance and use of fluorine was to be determined.

**Materials and Methods:**

The study lasted 15 months and was conducted from April 2018 to July 2019: an anonymous 29-question questionnaire was administered to all parents who accompanied their children (aged between 3 and 12 years) going under treatment in the Pediatric Dentistry Unit of the University Hospital Policlinico Umberto I, Rome. Anamnestic data, sociodemographic context (e.g., educational level and occupation), oral health habits, and prevention of parents and children and fluoride knowledge were investigated. The study received ethical approval. 204 questionnaires were collected. The data gathered were recorded with a specifically designed computer program and collected and analyzed using a Microsoft Excel 10 database. Data were evaluated using standard statistical analysis software; descriptive statistics including mean ± SD values and percentage were calculated for each variable. The relationship between the age of parents, between mother or father and the parents' degree of education levels, and the knowledge for their own children's oral health was explored using the chi-square test of homogeneity and Fisher's exact test (*P* value of < 0.05 considered as statistically significant).

**Results:**

From the acquired data, it is possible to deduce that the major respondents were mothers aged from 36 to 45, while only a small part were fathers aged above 45 years. Questions related to parents' oral hygiene habits were included in the questionnaire, and from the sample taken into consideration, it emerges that 64.7% of the respondents (67.1% mothers and 57.7% fathers) periodically attend a dental office for a checkup, 20.9% tend to postpone the treatment, and 15.2% go there just for emergency. Some of the questions showed that 80% of the interviewed subjects use fluoride toothpaste for their child's oral hygiene.

**Conclusion:**

Prevention in childhood, in addition to being synonymous with monitoring the oral health of the child, means first of all to pay attention to parents who are the main behavioral reference. It emerged that there is no adequate knowledge about fluorine, especially when the subjects have a low educational level. A role of fundamental importance for the diffusion of adequate concepts in the field of oral hygiene is covered, according to the data received from the study carried out, by the dentist and dental hygienist.

## 1. Introduction

The industrialization of many countries has led to an increase in chronic degenerative diseases [1], which are the consequence of many behavioral factors and lifestyles indirectly imposed by the society for years [2]. In healthcare, therefore, the need to pay more attention to the achievement of two objectives within the society arises: health promotion and prevention in terms of nutrition, good education, sport, and health education. Even though dental caries significantly decreased in western countries, it is still considered one of the main public health problems affecting most of the preschool children in many countries worldwide in the form of early childhood caries (ECC) [3].

Dental caries is a multifactorial disease that starts with microbiological changes within the complex biofilm and is affected by salivary flow and composition, exposure to fluoride, consumption of dietary sugars, etc. This affects humans of all ages all over the world and remains a major dental health problem among schoolchildren globally. [3]

The prevalence of ECC ranged from 1 to 12% in children living in developed countries [4]. The crucial reason for this situation is mainly ascribable to parents' or caregivers' lack of awareness of the potential disease [5]. Scientific evidence shows that adequate health standards must be learned since childhood through the help of parents [6] and appropriate school projects [7, 8].

Therefore, parental intervention must be appropriate to support the responsibility of their child's health. In oral health, it has been established for many years that there is a correlation between parental behaviors and lifestyle and children's attitude [5, 9]. It has also been established that the trend of the social and economic level of the family unit is also closely and proportionally to the interest of oral health itself [10]. Pediatricians' awareness regarding the process of dental caries is essential, as well as its prevention through early dental visits and available interventions, including fluorine [11]. The mechanisms of fluorine action are both topical and systemic, but the topical effect is the most important one. Fluorine has three main mechanisms of action: it reduces enamel demineralization; it promotes enamel remineralization; and it inhibits bacterial metabolism and acid production [12].

For this reason, this study aims to verify the close relation between behaviors, habits, lifestyles, and the knowledge of parents about their oral health and, consequently, the attention for their own children's oral health. In addition to this comparison, the second aim was to determine the degree of knowledge of parents about the importance of fluorine, whether they used fluoride products for the domestic oral hygiene of their children and their satisfaction about this choice.

## 2. Materials and Methods

The study was conducted from April 2018 to July 2019, and an anonymous questionnaire was administered to all parents who accompanied their children (aged between 3 and 12 years) going under treatment in the Pediatric Dentistry Unit of the University Hospital Policlinico Umberto I, Rome. The questionnaire validation was verified in a preliminary study [13].

The drafting of the questionnaire is derived from the analysis and subsequent combination of several scientifically validated questionnaires that have contributed over the years to determine the concept and importance of an individual's health:

- The HU-DBI questionnaire, Hiroshima University Dental Behavioral Inventory for the description of habits in oral health [14]
- The EGOHID questionnaire derived from a European project of development of oral health indicators [15]
- The TPB questionnaire theory of planned behavior [16]
- The MHLC questionnaire, multidimensional health locus of control [17]

The final version of the questionnaire included a total of 29 questions which have been divided into four sections, to make it easier to understand.

The first section corresponded to the collection of anamnestic data (parental figures, nationality, age, province of residence, number, and age of children in the family) and data related to the sociodemographic context of the interviewed subjects (educational qualification and profession). Particularly, the educational qualification was assessed dividing it into the categories elementary school, middle school, high school, and degree, while the categories specified for the education part were manager/entrepreneur, freelance, employee, workman, housewife, student, unemployed, and others. This information helps to have a generic but complete picture of the physiological and economic-social aspects of the subject. The second section included questions related to the attention given to their oral health and prevention. The third section was completely focused on the habits and behaviors adopted by the children for oral hygiene. The fourth and last sections, on the other hand, were dedicated to fluoride, testing the parents' knowledge on this topic and the source of information acquired.

The inclusion criteria were the age of the children between 3 and 12 years old and that the questionnaire had to be completed in each part.

The study protocol complied with the Ethical Guidelines of the 1975 Declaration of Helsinki and was approved by the ethics committee of Sapienza University of Rome.

The questionnaire included an informed consent to be signed, and this was obtained from all subjects participating in the study.

Three researchers took care of the creation of the manuscript, its administration and the collection of the data and results, while another one focused and developed the descriptive and statistical analysis.

### 2.1. Statistical Analysis

204 questionnaires were collected, each one of them properly filled, and with children within the age range; therefore, none of them was excluded. The data gathered through the questionnaire were recorded with a specifically designed computer program and collected and analyzed using a Microsoft Excel 10 database. Data were evaluated using standard statistical analysis software (version 20.0, Statistical Package for the Social Sciences, IBM Corporation, Armonk, NY, USA). Descriptive statistics including mean ± SD values and percentage were calculated for each variable. The relationship between the age of parents, between mother or father and the parents' degree of education levels, and the knowledge for their own children's oral health was explored using the chi-square test of homogeneity and Fisher's exact test. A *P* value of < 0.05 was considered as statistically significant.

## 3. Results

This trial collected 204 questionnaires completed by parents interviewed at the Pediatric Dentistry Unit of the University Hospital Policlinico Umberto I, Rome.

The medical history and sociodemographic characteristics of the sample are shown in Table 1.

From the acquired data, it is possible to deduce that the major respondents were mothers (74) aged from 36 to 45 and over 45 (56), while the remaining only 52 were fathers aged mainly between 36 and 45 or over 45.

The percentages of the sociocultural level, deduced from the qualification, were unchanged between the two parental figures as shown in Figure 1.

Questions related to parents' oral hygiene habits were included in the questionnaire, and from the sample taken into consideration, it emerges that 64.7% of the respondents (67.1% among all the mothers and 57.7% among all the fathers) periodically attend a dental office for a checkup, 20.9% tend to postpone the treatment, and 15.2% go there just for emergency.

To the question “How often do you usually attend a dental practice?”, the prevailing answer was “Periodically, even just for a check” (64.7% of the total interviewees, 67.1% among all the mothers, and 57.7% among all the fathers), followed by “Periodically, but in case of problems that are not very relevant to me, I tend to postpone the treatment” (20.9% of the total respondents, 19.07% of whom are mothers, and 23.07% of the fathers) and finally “Only in cases of emergency, for example in the presence of pain” (15.19% of the total interviewees, 13.81% from mothers, and 19.23% from fathers). When questioned if “Don't the baby's milk teeth need a good cure because they will fall anyway?”, a consistent result was found: 87.8% of the interviewed subjects did not agree, 7.3% were uncertain, and finally, 4.9% agreed not to perform treatment.

While in the previous question, there was a similar percentage of responses between the two parental figures, in this case, 90.1% of mothers think that it is important to care of deciduous teeth, while for the fathers, the percentage was 78%.

Regarding the attitude to the oral hygiene care of the child, the questions and percentages of the respective answers are shown in Table 2.

Some of the previous questions showed that 80% of the interviewed subjects use fluoride toothpaste for their child's oral hygiene: of this, 80%, 57% declare to choose the toothpaste to prevent the onset of dental caries (and is therefore aware of the benefits of fluorine), while the remaining 43% buys fluoride toothpastes for reasons other than the ultimate end of the fluorine itself (and is therefore not aware of its action).

Referring to the last section of the questionnaire, of the 204 people interviewed, 52.4% are aware of information related to fluorine, while the remaining 47.6% say they have no notion about fluorine itself.

The sources from which the subjects learn fluorine notions more or less effectively are represented in Figure 2.

The subjects who said they were informed about this topic were asked which is, in their opinion, the role of the fluoride contained in the toothpaste. The results are shown in Table 3.

It is possible to observe how 81.28% (row 1 of Table 3), or almost all subjects who declared to be aware of the role of fluorine, know exactly what the action of this element is, while a much lower percentage (18.72%) believes he knows it (rows 2 and 3 of Table 3), but in reality, does not. More specifically, we can see that the quantity of outliers is much lower if the information about fluorine is provided by the dental hygienist or dentist, and we can deduce that the role of these professionals is much more effective than other tools in the diffusion and in learning about the role and effectiveness of this element.

Furthermore, the part of the sample that uses fluoridated products for the oral hygiene of their children has been asked whether they are satisfied with their use and, if not, to motivate their cause: 90.8% of their parents are satisfied, while 9.2% say they are not because the dental caries have appeared the same even if much attention has been paid to oral hygiene.

To deepen the analysis, we asked to use that part of the sample that used fluoridated products (80%) if

- they use both toothpaste with fluorine and a mouthwash with fluorine or only one of the two
- for the type of fluoride product used, the concentration of fluorine is to be respected according to the age of the child

These results are shown in percentage values in Figures 3 and 4.

In support of the good knowledge about the role of fluoride by the parents highlighted above, these two figures illustrate how the parenting culture about this topic is reflected also in children.

Regarding the prevention of the carious lesion, as well as the use of topical fluoride, much importance has also been placed on the execution of dental sealants in T developmental age, for which the last three questions of the questionnaire are reserved.

67.15% of the interviewed subjects know what the dental sealants are, while the remaining 32.85% are not aware of the information in this regard: more in detail, from the statistically elaborated data, it emerges that the knowledge of dental sealants is greater in mothers (71.71%) compared to fathers (53.84%).

In addition, 162 questionnaires were selected out of a total of 204 that correspond to 162 parents with children aged between 6 and 12 years (that is, the age group in which the first permanent dental elements erupt as this performance it must be performed starting from these categories of teeth): to the question “Have your child ever had dental sealings done?”, the answers were affirmative for 41.97% of which the totality proved to be satisfied (unlike the degree of satisfaction of the use of fluoridate products for which some respondents have responded negatively) and negative for 43.82%, and the remaining 14.19% of parents do not even know if they have ever had them done to their children.

Regarding the knowledge of children's oral health, no difference was found correlating it with the age of the parents (*P* = 0.923), between mother and father (*P* = 0.293) and the parents' educational level (*P* = 0.817).

## 4. Discussion

From the statistical results obtained through the processing of the information collected, it was possible to make comparisons, setting variables, to compare what emerges from this study and what is evident from numerous studies conducted in literature with the same method, or data collection through the compilation of paper questionnaires by parents.

As already demonstrated by many articles in literature [5, 10, 18–20], the importance of oral care is often transmitted from parent to child with the same attitudes and attention that parents apply to themselves. For this reason, questions related to parents' oral hygiene habits were included in the questionnaire, and from the sample taken into consideration, it emerges that 64.7% of the respondents (67.1% mothers and 57.7% fathers) attend a dental office periodically for a check, 20.9% tend to postpone the treatment, and 15.2% just for emergency.

By grouping the different educational levels of the parents into two groups (the first of which is composed by elementary and lower secondary school certificate and the second by upper secondary school and graduates), it emerges that there is a considerable difference regarding the acquisition of fluoride notions: the first band, composed of 32 subjects, is equally balanced between subjects who are correctly informed about the role of fluorine and not; on the contrary, in the second band, which includes 172 subjects with a medium-high educational level, it is found that 70% of the subjects are correctly informed, while 30% do not have the right notions on this element.

This finding is also supported by other studies, in which the knowledge and attitude of the parents on oral health were assessed stating that subjects with higher educational level have greater knowledge about the topic [11–14, 21, 22].

Regarding one of the studies mentioned above and conducted in Greater Noida, it is stated that the knowledge and attitude of the parents does not vary significantly with age as putting two group variables: parents aged under 25 and parents aged 26 or over [21].

The other way around, in this study, if on the one hand, it is true that different age groups were taken into consideration (even if not by much compared to the study conducted in Greater Noida), on the other, it is true that differences have been found: indeed, subdividing the respondents in subjects aged 35 years or less and those aged 36 or over, 47.82% of parents in the first age group has good knowledge about the role of fluorine, while up to 69% among subjects aged 36 or over, noting that in addition to the educational level is also the age of the subject to influence on the knowledge of this information.

In a study published in the Evidence-Based Dentistry database by Topping and Assaf, it has been observed that when the child brushes his teeth alone, parental supervision helps to reduce the occurrence of caries more than when such supervision is not carried out. Furthermore, it emerges that parents who do not exercise direct control over their child's oral hygiene at home and who are not very present in daily household activities due to work commitment are less aware of the importance of brushing and the use of fluoride toothpastes [23].

To be able whether to sustain this phenomenon or not, data from the abovementioned study [23] were compared with the results of our trial: out of 204 interviewed subjects, 74.5% said that their child clean their teeth by himself. When asked “While the child is brushing his teeth, is there anyone looking at him?”, 8.55% say they do not control their child because they do not have time due to work commitments. Even if the percentage of those who do not supervise their children is very small, it is important to analyze how many of them know fluoride or not: of that 8.55%, only 15.4% say they are informed about the importance of fluorine itself, while the remaining 84.6% state the opposite; some of them declare that they have no specific reasons for choosing a toothpaste or using what they have at home for their children. In agreement with what has been deduced from the study of Topping and Assaf, it is also possible to affirm that parents who do not assist their children and who are not present in the routine of daily actions or who do not adopt direct control are uninformed about the importance of supervision and notions about fluorine, not considering the choice of toothpaste type as important.

In relation to what has been reported in this study and in the numerous scientific articles cited above regarding the positive effect of the educational level in the prevention of caries lesions, the mother's attitude and knowledge about oral health appears to be of considerable importance as they are statistically more present and they deal more frequently with their children's oral hygiene.

To support this data, together with the aim of understanding if there is a relationship between the strong incidence of caries (in 2010, it was found that 45% of children aged 5 years were affected by caries) and the behavior of parents about oral health, there is a study conducted in the Czech Republic. This study compares the positive effects that can be derived from the high educational levels of the mother with those of the father, asserting that the latter does not determine a significant influence on the oral health of the child as it is the mother, statistically, to take responsibility for the oral healthcare of the child himself [24]. Lencova and Duskova took the mid-high educational level of the parents (all parents who have acquired the high school diploma and the degree title) as the reference variable to verify, firstly, the percentage of mothers and fathers that really knew about fluorine and, secondly, if the awareness of mothers is actually more decisive and effective. Regarding the first hypothesis, 70% of mothers and 68% of fathers are correctly informed: as already stated above, the subjects with an adequate educational level are more aware about oral health, and in this case, there is no significant percentage difference between the two parental figures. Regarding the second hypothesis, it is possible to state that the awareness about oral health and the use of fluorine is more decisive in the education of the child if it is acquired by the mother, since the data processing shows that mothers are the parental figure that more frequently accompanies their children to various dental appointments. This phenomenon can be derived from the employment status as 30% of mothers are housewives or unemployed, while all paternal figures in the totality of the sample carry out a profession that does not allow a strong presence in everyday life. Precisely for these reasons, statistically, it is the mother, the main responsible for the oral health of the child and consequently having more time to devote to it, more frequently making decisions for him. In support of the argument, just exposed emerge from further statistical questionnaires about it: in fact, 25.5% of parents that claimed to brush himself their child's teeth consisted of 4 fathers and 48 mothers.

Within the prevention methods, dental sealants play an important role in preventing the onset and the development of dental cavities and became a worldwide prevention measure in the last decades [25, 26]. According to literature, mothers more than fathers have a positive opinion about dental sealants and that there is greater satisfaction with the use of fluoride products in larger families [19]. In the present study, it emerges that 67.15% of the subjects know what dental sealants are, of which 79.6% are mothers and the remaining 20.4% are fathers. Contrary to what emerges in the literature, both mothers and fathers are satisfied about the use of this benefit.

Regarding the use of fluorinated products, mouthwashes are a very popular additional oral hygiene element [27, 28], and in our study, a good percentage was found to use them together with a fluoride toothpaste, with high satisfaction regarding it.

## 5. Conclusions

From the ministerial guidelines, resulting from the November 2013 referred to the 2008 document, it was stated that “The individual risk of developing caries lesions should be evaluated through the experience of caries, dietary habits and oral hygiene, fluoride and the general state of health of each individual, as well as through the socio-economic status of the family” [29].

These factors can be assessed by studying the importance that the parent gives to oral healthcare, health education that will transmit to the child, and the attitudes about their oral hygiene at home. The elaboration of the data obtained from this study allowed to have a lot of information about these problems, crossing some variables among them.

It emerged, in fact, that most of the interviewees use fluoride products for the hygiene of their children, but only a part of these is aware of the positive effects that this has about the prevention of caries lesions: there is not adequate knowledge about fluorine, especially when the subjects have a low educational level.

The study also shows that mothers pay more attention and care to their children's oral health than fathers: the study shows that, if the educational level of the parents is medium-high, education related to oral hygiene will be more effective if it is given by the mother that is also considered the parental figure most available to perform performance to prevent the onset of carious lesions.

Moreover, age influences the acquisition of concepts, assuming that, if the subject understands the importance of prevention, with the passing of the years, he is increasingly determined to know as much information as possible for the maintenance of good oral health.

Even if minimal, a part of the interviewed subjects does not place the right importance on contemporary or subsequent brushing supervision if their child is autonomous in the management of oral hygiene: nonsupervision has also been synonymous with superficiality and less awareness. Therefore, prevention in childhood, in addition to being synonymous with monitoring the oral health of the child, means first of all to pay attention to parents who are the main behavioral reference model since the learning and adoption of good habits during childhood begins and is learned at home with the parental figures: a role of fundamental importance for the diffusion of adequate concepts in the field of oral hygiene is covered, according to the data received from the study carried out, by the dentist and dental hygienist.

## Figures and Tables

**Figure 1:** Sociocultural level, in percentage, of the interviewed subjects.

**Figure 2:** Sources from which the acquired information is derived.

**Figure 3:** Fluorine products used for the child.

**Figure 4:** Type of fluoride products used for children, under the age of 6 years.

**Table 1:** Medical history and sociodemographic characteristics of the sample.

Anamnestic and socio-demographic characteristics	Mother	Father	Total
N.	152 (74.5%)	52 (25.5%)	204
Nationality			
Italian	138 (90.7%)	49 (94.23%)	187 (91.6%)
Other	14 (9.2%)	3 (5.76%)	17 (8.3%)
Province			
Roma	126 (83%)	48 (92.23%)	174 (85.29%)
Viterbo	3 (2%)	0	3 (1.47%)
Latina	5 (3%)	2 (3.84%)	7 (3.43%)
Frosinone	11 (7.3%)	1 (1.92%)	12 (5.88%)
Rieti	3 (2%)	1 (1.92%)	4 (1.96%)
Other	4 (2.6%)	0	4 (1.96%)
Age			
Up to 29 years	10 (6.5%)	1 (1.92%)	11 (5.39%)
30-35 years	12 (8%)	0	12 (5.88%)
36-45years	74 (48.6%)	21 (40.38%)	95 (46.56%)
Over 45 years	56 (37%)	30 (57.69%)	86 (42.15%)
Education			
Primary school	4 (2.6%)	1 (1.92%)	5 (2.45%)
Middle school	21 (13.8%)	6 (11.53%)	27 (13.23%)
Upper secondary school	73 (48%)	25 (48.07%)	98 (48.03%)
Graduation	54 (35.6%)	20 (38.46%)	74 (36.27%)
Occupation			
Manager/businessman	4 (2.6%)	2 (3.84%)	6 (2.94%)
Free professional	16 (10.5%)	8 (15.38%)	24 (11.76%)
Employed/self-employed	68 (45%)	33 (63.5%)	101 (49.5%)
Worker	15 (9.8%)	8 (15.8%)	23 (11.27%)
Housewife	33 (21.71%)	0	33 (16.17%)
Student	4 (2.7%)	1 (1.9%)	5 (2.45%)
Unemployed	12 (7.8%)	0	12 (5.88%)
Other	0	0	0
N. of children in the family			
1			53 (25.98%)
2-3			137 (67.15%)
4-5			14 (6.86%)

**Table 2:** Child's attitude to oral hygiene care.

Child's attitude to oral hygiene care	Percentage
When did you start cleaning your child's teeth?	
a. Immediately after the first milky tooth eruption	32.8%
b. After the eruption of 4-6 teeth	34.31%
c. After the eruption of all the teeth	19.11%
d. I do not remember	13.72%
What do you use to clean your child's teeth?	
a. Finger	1.47%
b. Gauze	0.49%
c. Toothbrush	97.05%
d. I just rinse the mouth after meals	1%
Which substance do you use during teeth cleaning?	
a. Fluoride toothpaste	80%
b. Nonfluoride toothpaste	18.6%
c. Water	1.47%
d. Other	0
How many times?	
a. 3 times a day (after 3 meals)	22.05%
b. 2 times a day (morning and evening)	62.7%
c. 1 time a day	12.7%
d. Only sometimes a week	2.45%
In everyday life, who cleans the child's teeth?	
a. Mother	23.03%
b. Father	1.96%
c. Somebody else	0.5%
d. The child cleans the teeth by himself (go to the next question)	74.5%
While the child is brushing his teeth, is there anyone looking at him?	
a. Yes, even if he was well educated on the right movements to be done	36.84%
b. There is no one with him, but later, I check if he has brushed his teeth	54.60%
c. No control because no one in the family has time due to daily commitments	8.55%
When does he/she eat sugary food products?	
a. Together with meals	17.94%
b. Between meals during the day	81.86%
c. Before going to sleep to facilitate sleep	0.5%
Based on what do you choose the toothpaste for your child?	
a. Prevention of the onset of dental caries	58%
b. Prevention of gingival inflammation	5%
c. Prevention of bad breath	1.9%
d. Depending on the design of the container or the color	0.9%
e. A good taste of toothpaste	13.2%
f. What we have at home	7.8%
g. I have no specific reasons for choosing toothpaste	13.2%

**Table 3:** Percentage of the responses of the subjects informed on the basis of the information source.

	From ministry's guidelines	From dentist or dental hygienist	From the advertisement	From friends or acquaintance
Prevents the onset of dental caries	7.47%	57%	9.34%	7.47%
Prevents gum problems	1.86%	3.73%	0	0
It gives a sense of freshness	0.93%	5.69%	2.79%	3.72%

## Data Availability

Data are available upon request to the corresponding author.

## References

[1] Bontà G., Campus G., Strohmenger L., Cagetti M. G. (2018). Role of sugars and other sweeteners in the maintenance of the dental health. *Dental Cadmos*.

[2] World Health Organization (2005). *Preventing chronic diseases: a vital investement*.

[3] Jain M., Namdev R., Bodh M., Dutta S., Singhal P., Kumar A. (2015). Social and behavioral determinants for early childhood caries among preschool children in India. *Journal of Dental Research, Dental Clinics, Dental Prospects*.

[4] Colak H., Dülgergil C. T., Dalli M., Hamidi M. M. (2013). Early childhood caries update: a review of causes, diagnoses, and treatments. *Journal of Natural Science, Biology, and Medicine*.

[5] Vozza I., Capasso F., Marrese E., Polimeni A., Ottolenghi L. (2017). Infant and child oral health risk status correlated to behavioral habits of parents or caregivers: a survey in Central Italy. *Journal of International Society of Preventive & Community Dentistry*.

[6] Hamilton K., Cornish S., Kirkpatrick A., Kroon J., Schwarzer R. (2018). Parental supervision for their children's toothbrushing: mediating effects of planning, self-efficacy, and action control. *British Journal of Health Psychology*.

[7] Vozza I., Guerra F., Marchionne M., Bove E., Corridore D., Ottolenghi L. (2014). A multimedia oral health promoting project in primary schools in Central Italy. *Annali di Stomatologia*.

[8] Vozza I., Capasso F., Calcagnile F. (2019). School-age dental screening: oral health and eating habits. *Clinica Terapeutica*.

[9] Finlayson T. L., Siefert K., Ismail A. I., Sohn W. (2007). Maternal self-efficacy and 1?5-year-old children's brushing habits. *Community Dentistry and Oral Epidemiology*.

[10] Feldens C. A., Fortuna M. J., Kramer P. F., Ardenghi T. M., Vítolo M. R., Chaffee B. W. (2018). Family health strategy associated with increased dental visitation among preschool children in Brazil. *International Journal of Paediatric Dentistry*.

[11] Mahat G., Bowen F. (2017). Parental knowledge about urban preschool children’s oral health risk. *Pediatric Nursing*.

[12] Clark M. B., Slayton R. L., Section on Oral Health (2014). Fluoride use in caries prevention in the primary care setting. *Pediatrics*.

[13] Tranquilli M. (2018). *Experimental Study about the Awareness of Fluorine Importance in the Evolutive Age, [Ph.D thesis]*.

[14] Komabayashi T., Kwan S. Y., Hu D. Y., Kajiwara K., Sasahara H., Kawamura M. (2005). A comparative study of oral health attitudes and behaviour using the Hiroshima University-Dental Behavioural Inventory (HU-DBI) between dental students in Britain and China. *Journal of Oral Science*.

[15] Bourgeois D. M., Christensen L. B., Ottolenghi L., Llodre J. C., Pitts N. B., Senakola E. (2008). *Health surveillance in Europe. European Global Oral Health Indicators Development Project. Oral Health interviews and clinical surveys: Guidelines*.

[16] Ajzen (2002). *Theory of planned behaviour*.

[17] Wallston K. A., Wallston B. S., DeVellis R. (1978). Development of the multidimensional health locus of control (MHLC) scales. *Health Education Monographs*.

[18] Calcagnile F., Pietrunti D., Pranno N., Di Giorgio G., Ottolenghi L., Vozza I. (2019). Oral health knowledge in pre-school children: a survey among parents in Central Italy. *Journal of Clinical and Experimental Dentistry*.

[19] Blumer S., Ratson T., Peretz B. (2018). Parents’ attitude towards the use of fluorides and fissure sealants and its effect on their children’s oral health. *The Journal of Clinical Pediatric Dentistry*.

[20] Luzzi V., Ierardo G., Corridore D. (2017). Evaluation of the orthodontic treatment need in a paediatric sample from Southern Italy and its importance among paediatricians for improving oral health in pediatric dentistry. *Journal of Clinical and Experimental Dentistry*.

[21] Sehrawat P., Shivlingesh K. K., Gupta B., Anand R., Sharma A., Chaudhry M. (2016). Oral health knowledge, awareness and associated practices of pre-school children’s mothers in Greater Noida, India. *The Nigerian Postgraduate Medical Journal*.

[22] Elkarmi R., Shore E., O’Connell A. (2015). Knowledge and behaviour of parents in relation to the oral and dental health of children aged 4-6 years. *European Archives of Paediatric Dentistry*.

[23] Topping G., Assaf A. (2005). Strong evidence that daily use of fluoride toothpaste prevents caries. *Evidence-Based Dentistry*.

[24] Lencova E., Duskova J. (2013). Oral health attitudes and caries-preventive behaviour of Czech parents of preschool children. *Acta Medica Academica*.

[25] Colombo S., Paglia L. (2018). Dental sealants. Part 1: prevention first. *European Journal of Paediatric Dentistry*.

[26] Wright J. T., Tampi M. P., Graham L. (2016). Sealants for preventing and arresting pit-and-fissure occlusal caries in primary and permanent molars: a systematic review of randomized controlled trials-a report of the American Dental Association and the American Academy of pediatric dentistry. *Journal of the American Dental Association (1939)*.

[27] Radzki D., Wilhelm-Węglarz M., Pruska K., Kusiak A., Ordyniec-Kwaśnica I. (2022). A fresh look at mouthwashes-what is inside and what is it for?. *International Journal of Environmental Research and Public Health*.

[28] Pilli L. N., Singaraju G. S., Nettam V., Keerthipati T., Mandava P., Marya A. (2022). An extensive comparison of the clinical efficiency of acidulated phosphate fluoride (APF) and neutral sodium fluoride (NaF) oral rinses in the prevention of white spot lesions during fixed orthodontic treatment: a randomized controlled trial. *BioMed Research International*.

[29] Italian Health Minister (2013). *National Guidelines for the oral heath prevention and prevention of oral pathologies in developmental age*.

